RETRACTED

# m^6^A modification-mediated CBX8 induction regulates stemness and chemosensitivity of colon cancer via upregulation of LGR5

**DOI:** 10.1186/s12943-019-1116-x

**Published:** 2019-12-18

**Authors:** Yi Zhang, Min Kang, Bin Zhang, Fanchao Meng, Jun Song, Hiroshi Kaneko, Fumio Shimamoto, Bo Tang

**Affiliations:** 1 Department of Health Sciences, Hiroshima Shudo University, 1-1-1, Ozuka-higashi, Asaminami-ku, Hiroshima, 731-3195 Japan; 2 Department of General Surgery, Affiliated hospital of Xuzhou Medical University, Xuzhou, 221000 China; 3 Department of Obstetrics, Gynecology and Reproductive Sciences, Yale School of Medicine, New Haven, CT 06510 USA; 4 Department of Oncology, The First Affiliated Hospital of Dalian Medical University, Dalian, 116011 China

**Keywords:** Colon cancer, Cancer stemness, m^6^A, CBX8

## Abstract

**Background:**

Colon cancer (CC) cells can exhibit stemness and expansion capabilities, which contribute to resistance to conventional chemotherapies. Aberrant expression of CBX8 has been identified in many types of cancer, but the cause of this aberrant CBX8 expression and whether CBX8 is associated with stemness properties in CC remain unknown.

**Methods:**

qRT-PCR and IHC were applied to examine CBX8 levels in normal and chemoresistant CC tissues. Cancer cell stemness and chemosensitivity were evaluated by spheroid formation, colony formation, Western blot and flow cytometry assays. RNA-seq combined with ChIP-seq was used to identify target genes, and ChIP, IP and dual luciferase reporter assays were applied to explore the underlying mechanisms.

**Results:**

CBX8 was significantly overexpressed in chemoresistant CC tissues. In addition, CBX8 could promote stemness and suppress chemosensitivity through LGR5. Mechanistic studies revealed that CBX8 activate the transcription of LGR5 in a noncanonical manner with assistance of Pol II. CBX8 recruited KMT2b to the LGR5 promoter, which maintained H3K4me3 status to promote LGR5 expression. Moreover, m^6^A methylation participated in the upregulation of CBX8 by maintaining CBX8 mRNA stability.

**Conclusions:**

Upon m^6^A methylation-induced upregulation, CBX8 interacts with KMT2b and Pol II to promote LGR5 expression in a noncanonical manner, which contributes to increased cancer stemness and decreased chemosensitivity in CC. This study provides potential new therapeutic targets and valuable prognostic markers for CC.

## Background

Colon cancer (CC) is a leading cause of cancer-related death in many countries [1]. Therefore, the mechanisms underlying CC development need to be fully elucidated. Accumulating evidence has demonstrated that a distinct tumor cell subpopulation with stemness, known as the cancer stem cell (CSC) population, exists in CC [2]. CSCs can self-renew and expand, thus contributing to progression of tumors and resistance to conventional therapies [3]. Therefore, clarification of the detailed mechanism of CSC reprogramming is urgently needed and may suggest a promising strategy for overcoming CC chemoresistance.

RETRACTED

CBX8, also known as Human Polycomb 3, belongs to the CBX protein family (which includes CBX2, CBX4, CBX6, CBX7 and CBX8). The functions of CBX8 are complicated, and previous studies have suggested that CBX8 acts as an oncogene in certain types of cancer. For instance, CBX8 facilitates tumor growth and metastasis in hepatocellular carcinoma (HCC) [4] and breast cancer [5] and can induce tumor proliferation and inhibit tumor apoptosis in colorectal cancer (CRC) [6, 7]. However, whether CBX8 is associated with stemness properties and chemosensitivity remains unknown and needs further exploration in the context of CC.

Canonically, CBX8 is characterized as a transcriptional repressor that interacts with RING1a/b and BMI1 to construct Polycomb repressive complex 1 (PRC1) [8]. However, noncanonical roles of CBX8 in transcriptional regulation have also been documented. For example, CBX8 induces transcriptional activation in a PRC1-independent manner by interacting with MLL-AF9 and TIP60 [9]. In addition, CBX8 activates AKT/β-catenin signaling by upregulating the expression of the transcription factor EGR1 and the miRNA miR-365-3p independently of PRC1 [4]. These observations suggest that the exact roles of CBX8 in transcriptional regulation remain largely undefined.

In this study, we found that CBX8 is significantly overexpressed in chemoresistant CC tissues, suggesting that CBX8 may be involved in cancer stemness and chemosensitivity regulation. In vivo and in vitro experiments confirmed that CBX8 can promote the stemness properties of CC cells and suppresses the sensitivity to chemotherapy. Mechanistically, CBX8 can noncanonically bind to Pol II and recruit KMT2b, a histone H3 lysine 4 (H3K4) methyltransferase, to the LGR5 promoter and can sustain LGR5 gene expression by maintaining the status of the transcription-activating H3K4 trimethylation (H3K4me3) modification. Finally, aberrant overexpression of CBX8 in CC is caused by Mettl3-induced N6-methyladenosine (m^6^A) modification which maintains the stability of CBX8 mRNA.

## Methods

### Patient samples

This study was reviewed and approved by the Ethics Committee of the Affiliated Hospital of Xuzhou Medical University, and written informed consent was obtained from all patients. The study included 40 metastatic CC patients aged 30 to 80 years. All patients were treated with first-line Oxaliplatin-based chemotherapy, and 13 of them underwent surgery before or after chemotherapy between 2016 and 2018 at the Department of General Surgery. Chemotherapy responses were evaluated using the tumor regression grade (TRG) system. The patients were divided into two groups based on their response to chemotherapy: a chemoresistant (R) group and a chemosensitive (S) group.

RETRACTED

### Cell lines and cell culture

The CC cell lines used in this study were purchased from the American Type Culture Collection (ATCC). These cell lines included LoVo, SW620, SW480, DLD-1, Colo205, HT-29, HCT116 and NCM460. HT-29, DLD-1 and Colo205 cells were cultured in RPMI-1640 medium (Gibco, USA); LoVo cells were cultured in F-12 K medium (Gibco, USA); SW620 cells were cultured in L-15 medium (Gibco, USA); and SW480, NCM460, and HCT-116 cells were cultured in modified Eagle’s minimum essential medium (Gibco, USA). All media were supplemented with 10% fetal bovine serum (FBS) and 1% antibiotic/antimycotic solution (Biowest, Nuaille, France). All cell lines were cultured in 5% CO_2_ at 37 °C in incubators with 100% humidity.

### Cell transfection

Short interfering RNA (siRNA) sequences were directly synthesized (GenePharma, Shanghai, China). The full-length human CBX8, LGR5 and Mettl3 sequences were cloned into the pcDNA3.1 vector with or without a Flag- or HA-tag sequence (Invitrogen, Shanghai, China). The siRNA and pcDNA3.1 were transfected into cells using Lipofectamine 3000 (Invitrogen, Shanghai, China). Two days later, the cells were harvested for further experiments.

shRNAs were delivered by lentiviral infection with lentiviruses produced by transfection of 293 T cells with the vector pLKO.1. Cells infected with lentiviruses delivering scrambled shRNA (shScr) were used as negative control cells. The shRNA and siRNA sequences are listed in the Additional file 7.

### Spheroid formation assay

A total of 1000 CC cells were plated in ultralow attachment plates. The cells were cultured for 10 days in DMEM/F12 medium (Invitrogen, Shanghai, China) supplemented with 4 mg/mL insulin (Sigma, Shanghai, China), B27 (1:50, GIBCO, Shanghai, China), 20 ng/mL EGF (Sigma, Shanghai, China) and 20 ng/mL basic FGF (Sigma, Shanghai, China). For the serial passaging of primary spheres, these were collected, dissociated with trypsin, resuspended in DMEM/F12 medium with the above supplements, and plated to generate secondary spheroids. The number of spheres was counted under the microscope, and the data are expressed as the mean ± SD of triplicate wells within the same experiment.

### Chromatin immunoprecipitation (ChIP) and ChIP-sequencing

A ChIP assay was carried out using an EZ-ChIP™ Chromatin Immunoprecipitation Kit (Millipore, Bedford, MA, USA) following the manufacturer’s protocols. Briefly, 1% formaldehyde was used to crosslink proteins and DNA for 10 min. Cell lysates were sonicated to obtain DNA fragments, which were subjected to IP with primary antibodies or negative control IgG. Purified DNA was analyzed by qRT-PCR with SYBR Green Master Mix (Promega, Beijing, China). The relative enrichment values were calculated through normalization of the results to the input values and are expressed relative to the values obtained with normal IgG. The primers used are listed in the Additional file 7. ChIP libraries were prepared using ChIP DNA according to the BGISEQ-500ChIP-Seq library preparation protocol. In-depth whole-genome DNA sequencing was performed by R&S (Shanghai, China).

RETRACTED

### Immunohistochemistry (IHC), Western blot analysis, Colony formation, flow cytometry, co-immunoprecipitation (CoIP), quantitative real time RT-PCR (qRT-PCR), RNA immunoprecipitation (RIP), microarray analysis, gene set enrichment analysis (GSEA), in vivo tumor growth assay and mouse Xenograft tumor treatment model

Details are provided in the Additional file 7.

### Statistical analysis

All values are expressed as the mean ± standard deviation (SD). The significance of the differences was determined via one-way ANOVA or Student’s t-test. Spearman’s correlation coefficient was used to calculate the correlations between the two groups. Kaplan–Meier analysis was employed for survival analysis, and the differences in the survival probabilities were estimated using the log-rank test. *P* < 0.05 was considered to indicate statistical significance. The statistical analyses were performed using SPSS version 17.0 (SPSS, Inc.).

## Results

### CBX8 maintains the stemness properties of CC cells

We used The Cancer Genome Atlas (TCGA) and the Genotype-Tissue Expression (GTEx) database to analyze the mRNA expression profiles of CBX proteins in normal colon tissues (*n* = 349) and CC tissues (*n* = 275), finding that the expression of CBX2, CBX4 and CBX8 was significantly upregulated in CC tissues (Additional file 1: Figure S1A). Then, we investigated the levels of the abovementioned three molecules in chemoresistant CC tissues by IHC. Interestingly, CBX8 expression was higher in chemoresistant CC tissues than in normal tissues (Additional file 1: Figure S1B).

As chemoresistance is a key feature of cancer stemness, we investigated the effect of CBX8 on the stemness features of CC cells. We confirmed that CBX8 was overexpressed in CC cell lines relative to normal epithelial cell lines (Additional file 2: Figure S2A). Ectopic suppression of CBX8 reduced primary and secondary spheroid formation ability in CC cells compared with the control cells (Fig. 1a, b). Conversely, CBX8 overexpression enhanced primary and secondary spheroid formation ability (Fig. 1c). Stemness markers reported for CC include CD133, CD44, LGR5 and EpCAM [10–12]. We also examined the potential regulatory effect of CBX8 on the expression of stemness markers. Suppression of CBX8 significantly reduced the expression of CD133, LGR5, CD44 and EpCAM in CC cells (Fig. 1d). On the other hand, CBX8 overexpression significantly increased the expression of stemness markers in CC cells (Fig. 1d). We also performed flow cytometry to assess the populations of LGR5^high^ cancer cells. Depletion of CBX8 reduced the proportions of LGR5^high^ CC cells (Fig. 1e, f). Conversely, CBX8 overexpression increased the LGR5^high^ cell populations (Fig. 1g). The role of CBX8 in regulating the stemness properties of CC was further investigated via subcutaneous inoculation of cells into NOD/SCID mice. Mice injected with CBX8 knockdown DLD-1 and LoVo cells exhibited appreciably reduced tumor incidence relative to control mice (Fig. 1h-i, Additional file 2: Figure S2B). Then, mice were injected with DLD-1 cells with or without CBX8 depletion in a limited dilution series and tumor incidence was monitored. CBX8 knockdown led to a greater than 80% reduction of CSC frequency in vivo (Additional file 2: Figure S2C).

RETRACTED

**Fig. 1:** CBX8 maintains the stemness of CC cells. **a-c,** Representative images of sphere formation induced by the transfection of shCBX8 into DLD-1 and LoVo cells or the transfection of a CBX8 overexpression plasmid into SW480 cells. The surviving colonies were measured for the number of tumorspheres. **d,** The expression levels of CSC markers, including CD133, CD44, LGR5 and EpCAM, were examined in shCBX8-transfected CC cells and CBX8 overexpression plasmid-transfected CC cells by Western blotting. **e-g,** Flow cytometry was used to assess the percentage of LGR5^high^ cells in CC cells with CBX8 depletion or overexpression. **h-i,** Tumor formation in nude mice injected with shCBX8-transfected DLD-1 and LoVo cells (5 × 10^4^ cells per mouse). The incidence of tumor formation was monitored for 40 days. **j,** Sphere formation of sorted LGR5+ and LGR5- DLD-1 cells. Only the top 2% most brightly stained cells or the bottom 2% most dimly stained cells were selected as LGR5+ or LGR5- populations, respectively. **k,** Xenograft tumors derived from serial subcutaneous injections of sorted LGR5+ and LGR5- DLD-1 cells. **l-m,** Sorted LGR5+ cells and LGR5- cells were treated with L-OHP and CPT-11. Apoptotic rate was detected by double-stained for Annexin V and PI and analyzed by flow cytometry. Data are shown as the mean ± SD of three replicates (*, *P* < 0.05; **, *P* < 0.01)

As LGR5+ colon cancer cells serve as CSCs [10], we further address whether LGR5+ cells possess cancer stemness properties. we sorted LGR5+ and LGR5- subsets from DLD-1 cells with CBX8 overexpression using fluorescence-activated cell sorting (FACS). Compared to LGR5- cells, LGR5+ cells had higher mRNA levels of CBX8 and stemness markers (Additional file 2: Figure S2D). Spheroid formation assays revealed that LGR5+ cells exhibited stronger spheroid formation abilities than LGR5- cells (Fig. 1j, Additional file 2: Figure S2E). Xenograft tumor formation was observed in 5 of 5 and 3 of 5 animals when 1 × 10^5^ and 1 × 10^4^ sorted LGR5+ cells, were subcutaneously injected into nude mice, respectively (Fig. 1k). No tumor formation was observed when the same numbers of LGR5- cells were injected, while tumor formation was only observed in 2 of 5 nude mice when 1 × 10^6^ of LGR5- cells were injected (Fig. 1k). Oxaliplatin (L-OHP), a platinum-based chemotherapeutic, and Irinotecan (CPT-11), a camptothecin derivative, are widely used in clinics against CCs. Consistent with stemness characteristics, sorted LGR5+ cells displayed a stronger ability to resist apoptosis induced by L-OHP (10 μM) or CPT-11(10 μM) treatment compared to that of LGR5- cells (Fig. 1l, m).

RETRACTED

### CBX8 suppresses the chemosensitivity of CC cells to L-OHP and CPT-11

Because CBX8 depletion inhibits the stemness of CC cells, we next examined whether CBX8 could affect the chemosensitivity of CC cells. Ectopic suppression of CBX8 sensitized CC cells to L-OHP (10 μM) and CPT-11(10 μM), as reflected by reduced colony formation ability and increased apoptotic rate (Fig. 2a, b, e). However, overexpression of CBX8 had the opposite effect (Fig. 2c, d, f). The statistical analyses demonstrated that CBX8 depletion or overexpression had a synergistic, rather than an additive, effect with chemotherapeutic agents (Additional file 3: Figure S3A, B).

**Fig. 2:** CBX8 suppresses the chemosensitivity of CC Cells to L-OHP or CPT-11. **a-b,** Colony formation in shCBX8-transfected CC cells after treatment with L-OHP or CPT-11 a concentration of 10 μmol/L. **c-d,** Colony formation in CBX8 overexpression plasmid-transfected CC cells after treatment with L-OHP or CPT-11 a concentration of 10 μmol/L. **e-f,** Flow cytometry was used to assess the apoptotic rate of CBX8-silenced DLD-1 cells and CBX8-overexpressed SW480 cells when treated with L-OHP or CPT-11 a concentration of 10 μmol/L. **g,** Representative images of xenograft tumors in nude mice after different treatments. Vec or shCBX8 were injected intratumorally once per week for 4 weeks. L-OHP or CPT-11 were injected intraperitoneally twice per week for 4 weeks. The combination of shCBX8 with L-OHP or CPT-11 had stronger inhibitory effects on tumor growth. **h,** The tumor growth curves of each group of mice are summarized. **i,** The levels of CBX8 and caspase 3 expression were assessed by IHC in different groups. Data are shown as the mean ± SD of three replicates (*, *P* < 0.05; **, *P* < 0.01)

To further investigate whether CBX8 knockdown affects chemosensitivity, a xenograft tumor induced by subcutaneously injecting of DLD-1 cells was removed and cut into 1 mm^3^ pieces and subcutaneously implanted into nude mice. After one week, the nude mice were divided into 6 groups (*n* = 5 per group) and received an intratumoral injection of an empty vector (Vec) or lentiviral-shCBX8 (shCBX8), meanwhile, 4 of 6 groups received the combination of the intraperitoneal injection of L-OHP or CPT-11. The results indicated that silencing CBX8 expression yielded effective inhibition of tumor growth compared to the Vec groups (Fig. 2g, h). The combination of shCBX8 with L-OHP or CPT-11 had stronger inhibitory effect on tumor growth than that with any individual treatment (Fig. 2g, h). IHC result confirmed that the expression of CBX8 was suppressed by shCBX8 (Fig. 2i). Moreover, the combination of shCBX8 with L-OHP or CPT-11 led to more apoptosis than other group, as determined by caspase 3 staining (Fig. 2i). Taking together, these data demonstrated that virus-mediated CBX8 silencing increased the chemosensitivity of CC cells to L-OHP and CPT-11.

RETRACTED

### LGR5 is identified as a target of CBX8 and mediates the CBX8-induced stemness in CC cells

To assess the impact of CBX8 on gene expression, we performed genome-wide expression analysis in both control and CBX8-depleted cells and identified the differentially expressed genes. CBX8 depletion resulted in upregulation of 2234 genes and downregulation of 3410 genes (Fig. 3a). The GSEA analysis results showed that the differentially expressed gene sets were significantly related to stemness and cancer aggression (Fig. 3b). We then determined the genome-wide target sites of CBX8 in CC cells using a ChIP-seq approach and identified 22,917 peaks corresponding to 4575 RefSeq genes. CBX8 was preferentially distributed near the transcription start sites (TSSs) of genes (Additional file 4: Figure S4A). The Gene Ontology (GO) analysis results showed that the most significant biological functions of the CBX8-binding genes included positive regulation of transcription, Pol II regulatory region sequence-specific DNA binding, and transcription corepressor activity (Additional file 4: Figure S4B). Then, we investigated the overlapping gene sets between the differentially expressed genes after CBX8 knockdown and the ChIP-seq data and found that 46 upregulated genes were included in the set of CBX8 target genes, while 83 downregulated genes were included in the set of CBX8 target genes (Fig. 3c). Interestingly, we found that the stemness marker, LGR5, was in the set of 83 downregulated target genes. Therefore, we evaluated whether CBX8 promotes stemness through LGR5.

RETRACTED

**Fig. 3:** CBX8 regulates LGR5 transcription by interacting with Pol II in a noncanonical manner. **a,** The heatmap of the differentially expressed genes after CBX8 knockdown. **b,** GSEA showed that genes differentially expressed in response to CBX8 knockdown were enriched in gene sets significantly related to stemness and cancer aggression. **c,** The Venn diagram showing the numbers of overlapping genes between the set of genes differentially expressed by CBX8 knockdown and the set of target genes identified by ChIP-seq. **d,** Overview of the LGR5 promoter region with ChIP-seq data for CBX8 and Pol II in DLD-1 cells. **e,** The top five predicted CBX8-binding elements were obtained by de novo motif analysis using MEME software. **f,** Luciferase reporter genes driven by the − 1224/− 592 or − 591/267 fragments of the LGR5 promoter region were cotransfected with shCtrl or shCBX8 into DLD-1 and LoVo cells, and luciferase activity was measured after 48 h. The relative luciferase activity value in cells cotransfected with pRL-TK (− 591/267) and shCtrl was set to 100%. **g,** Luciferase reporter genes driven by the − 1224/− 592 or − 591/267 fragments of the LGR5 promoter region were cotransfected with the empty vector (vec) or the CBX8 overexpression pcDNA3.1 plasmid into SW480 cells, and luciferase activity was measured after 48 h. **h,** A schematic of the seven LGR5 promoter regions (1–7) analyzed for CBX8 binding affinity (*above*). Schematic representation of predicted CBX8 and KMT2b binding sites (*below*). **i,** ChIP-qPCR analysis was used to determine the binding affinity of CBX8 to seven LGR5 promoter regions in DLD-1 cells, showing that CBX8 bound to the CBS1-CBS4 regions in the LGR5 promoter. ChIP-qPCR with IgG was performed as the control. **j,** Western blot analysis of LGR5 expression in Pol II knockdown DLD-1 cells with or without overexpressing CBX8. **k-l,** CoIP was used to show the interaction between the CBX8 and Pol II proteins in DLD-1 cells. **m,** ChIP-qPCR analysis was used to assess the binding affinity of Pol II to the CBS1-CBS4 regions after CBX8 knockdown in DLD-1 cells. **n,** Western blot was used to determine the expression of Ring1b and LGR5 after silencing of Ring1b in DLD-1 cells. Data are shown as the mean ± SD of three replicates (*, *P* < 0.05; **, *P* < 0.01)

To further evaluate the effect of LGR5 on CBX8-mediated stemness properties, we transfected CBX8-silenced CC cells with an LGR5 overexpression plasmid. LGR5 overexpression restored the changes in stemness marker expression, spheroid formation ability and chemosensitivity to L-OHP and CPT-11 induced by CBX8 depletion (Additional file 4: Figure S4C-E). Conversely, LGR5 knockdown rescued the changes in stemness marker expression, spheroid formation ability and chemosensitivity induced by CBX8 overexpression (Additional file 4: Figure S4C-E). These results confirmed that CBX8 promotes cancer stemness and inhibits chemosensitivity through LGR5.

RETRACTED

### CBX8 regulates LGR5 transcription by interacting with pol II in a noncanonical manner

Next, we investigated the underlying mechanism by which CBX8 promotes LGR5 expression. The results of qRT-PCR confirmed that CBX8 depletion resulted in LGR5 suppression, while enforced CBX8 expression resulted in LGR5 overexpression (Additional file 2: Figure S2F, G), suggesting that CBX8 modulated LGR5 expression at transcriptional level. The ChIP-seq results showed that CBX8 was enriched at the promoter of LGR5 (Fig. 3d). Then, MEME motif analysis was used to identify the binding motif for CBX8. Fig. 3e shows the top five predicted motifs. Notably, the fourth motif was enriched in the LGR5 promoter and may play a crucial role in the transcriptional regulation of LGR5. To determine whether a CBX8-responsive region was present, we constructed three luciferase reporters containing different fragments of the LGR5 promoter. The results of luciferase reporter assays showed that CBX8 knockdown significantly reduced luciferase activity driven by the − 591/267 fragment (Fig. 3f), whereas CBX8 overexpression enhanced luciferase activity driven by this fragment (Fig. 3g). The activity driven by the − 1224/− 592 construct was not affected by changes in CBX8 expression (Fig. 3f, g). These results confirmed that the − 591/267 region of the CBX8 promoter contained CBX8-responsive sites. Then, we constructed seven pairs of primers targeting different regions of the LGR5 promoter (regions 1–7, Fig. 3h). Combined ChIP and qPCR analysis revealed that CBX8 bound to regions 2–5 (also referred to as CBX8 binding site (CBS) 1-CBS4, respectively) in the CBX8 promoter (Fig. 3i), which are included in the − 591/267 fragment.

As GO analysis of the CBX8-binding genes revealed enrichment for Pol II regulatory region sequence-specific DNA binding, we evaluated whether Pol II participates in CBX8-induced LGR5 activation. The Western blot assay results showed that Pol II knockdown suppressed LGR5 activation in DLD-1 cells with or without CBX8 overexpression (Fig. 3j). The ChIP-seq data indicated strong enrichment of Pol II in the LGR5 promoter (Fig. 3d), and the CoIP assay results showed that CBX8 bound Pol II in DLD-1 cells (Fig. 3k, l). We also knocked down or overexpressed CBX8 and performed ChIP-PCR assays. The results showed decreased occupancy of Pol II at CBS2 and CBS4 when CBX8 was knocked down (Fig. 3m). In contrast, increased occupancy of Pol II at CBS2 and CBS4 was found after CBX8 overexpression (Additional file 5: Figure S5A). We also investigated whether CBX8 promotes LGR5 transcription in a canonical PRC1-dependent manner. To this end, we knocked down Ring1b expression in DLD-1 cells, but Ring1b knockdown did not interfere with LGR5 expression (Fig. 3n), suggesting that CBX8-mediated LGR5 activation may occur independently of the canonical mechanism involving PRC1.

RETRACTED

### CBX8 maintains the H3K4me3 status at the LGR5 promoter by binding to KMT2b

To gain insight into the mechanism by which CBX8 regulates LGR5 expression, we used the University of California-Santa Cruz (UCSC) Genome Bioinformatics Site (http://genome.ucsc.edu/) to determine the presence or absence of histone modifications (H3K4me3, histone H3 lysine 27 trimethylation (H3K27me3), and H3K27 acetylation (H3K27Ac)) on the LGR5 promoter. H3K4me3 and H3K27Ac mark transcriptional activation, while H3K27me3 marks transcriptional suppression. We found high enrichment and overlap of H3K4me3 and H3K27me3 peaks (Fig. 4a). ChIP assays were used to further determine whether CBX8 regulates LGR5 through histone modifications. Interestingly, CBX8 loss and overexpression decreased and increased H3K4me3 at the LGR5 promoter, respectively (Fig. 4b, c), whereas CBX8 depletion did not change H3K27me3 or H3K27Ac (Additional file 5: Figure S5B, C). These data implied that H3K4me3 modification at the LGR5 promoter accounted for the CBX8-mediated activation of LGR5.

**Fig. 4:** CBX8 maintains the H3K4me3 status at the LGR5 promoter by binding to KMT2b. **a,** Overview of the LGR5 promoter region with ChIP-seq data from ENCODE for H3K27me3, H3K4me3 and H3K27Ac in HCT-116 cells and for KMT2b in HepG2 cells. **b,** ChIP-qPCR analysis identified enrichment of H3K3me3 in the CBS1-CBS4 regions after CBX8 knockdown in DLD-1 cells. ChIP-qPCR with IgG was performed as the control. **c,** ChIP-qPCR analysis identified enrichment of H3K3me3 in the CBS1-CBS4 regions after CBX8 overexpression in DLD-1 cells. ChIP-qPCR with IgG was performed as the control. **d,** The RNAi screen of KMT2s (KMT2A-G) showed that KMT2b siRNA significantly downregulated LGR5 mRNA levels in DLD-1 cells. **e,** Western blot analysis of LGR5 expression in KMT2b knockdown DLD-1 cells overexpressing CBX8. **f,** CoIP showed the interaction between the CBX8 and KMT2b proteins in DLD-1 cells. **g,** HEK293 cells were transfected with Flag-tagged CBX8 with or without HA-tagged KMT2b. Lysates were subjected to IP using anti-Flag and anti-HA antibodies. **h,** ChIP-qPCR analysis performed to determine the binding affinity of KMT2b to the seven LGR5 promoter regions in DLD-1 cells showed that CBX8 bound to the KBS1-KBS3 regions in the LGR5 promoter. ChIP-qPCR with IgG was performed as the control. **i,** ChIP-qPCR analysis was used to determine the binding affinity of KMT2b to the KBS1-KBS3 regions after CBX8 knockdown. **j,** ChIP-qPCR analysis showed the enrichment of CBX8 and H3K4me3 in the CBS1-CBS3 regions after KMT2b knockdown in DLD-1 cells. **k,** Schematics of the luciferase reporter gene constructs. **l,** The luciferase reporter gene constructs were cotransfected with shCBX8 or shCtrl into DLD-1 cells, and reporter gene activity was measured after 48 h by a dual luciferase assay. The relative value in DLD-1 cells cotransfected with pGL3 (− 1224/317) and shCtrl was set to 100%. **m,** The luciferase reporter gene constructs were cotransfected with the CBX8 overexpression plasmid or empty vector into DLD-1 cells, and reporter gene activity was measured after 48 h by dual luciferase assay. **n,** Schematic of the five Flag-CBX8 recombinant proteins (CB1-CB5). **o,** Plasmids encoding a Flag-tagged, CBX8 truncation mutant were transfected into DLD-1 cells, anti-Flag antibody was used to immunoprecipitate the bound proteins, and the KMT2b level in the immunoprecipitates was determined by Western blot. Data are shown as the mean ± SD of three replicates (*, *P* < 0.05; **, *P* < 0.01)

Recent studies have reported that CBX proteins function in cooperation with other proteins to promote epigenetic activation or silencing of gene expression [13, 14]. As Set1/Trithorax-type H3K4 methyltransferases catalyze H3K4 methylation [15], we utilized an RNA interference (RNAi) screening approach to identify potential H3K4 modifiers responsible for LGR5 regulation. Notably, depletion of KMT2b, but not other enzymes, decreased LGR5 expression (Fig. 4d). In addition, the ChIP-seq data from ENCODE showed that KMT2b was enriched in the LGR5 promoter (Fig. 4a). Therefore, we investigated whether KMT2b participates in CBX8-induced LGR5 activation. The Western blot assay results showed that KMT2b knockdown suppressed LGR5 activation induced by CBX8 overexpression (Fig. 4e). In addition, the CoIP assay results showed that CBX8 interacted with KMT2b reciprocally in DLD-1 cells (Fig. 4f). Interaction between CBX8 and KMT2b was identified by CoIP when these labeled proteins were co-expressed in HEK293 cells (Fig. 4g). To further evaluate the role of KMT2b in CBX8-mediated LGR5 expression, we re-examined the seven regions of the LGR5 promoter by ChIP-qPCR (Fig. 3h). The ChIP assay showed that KMT2b was significantly enriched in regions 3, 5 and 6 (also referred to as KMT2b binding site (KBS) 1, KBS2 and KBS3, respectively) (Fig. 4h). CBX8 knockdown decreased the occupancy of KMT2b at KBS1 and KBS2 (Fig. 4i), while KMT2b depletion suppressed the enrichment of KMT2b and H3K4me3 at KBS1 and KBS2 (Fig. 4j). These results suggest that CBX8 causes accumulation of KMT2b at KBS1 and KBS2 to maintain H3K4me3 modification status. To further confirm whether KBS1 and KBS2 are the key sites for promotion of LGR5 expression, we constructed several luciferase reporter gene plasmids containing various promoter regions with or without mutation of KBS1 and KBS2 (Fig. 4k). Compared with that of the empty vector control, the activity driven by both pGL3 (− 1224/317) promoters significantly decreased and increased upon CBX8 knockdown and overexpression, respectively (Fig. 4l and m). However, when KBS1 or KBS2 was mutated or when KBS2 was deleted, CBX8 knockdown and overexpression decreased and increased reporter gene activity, respectively (Fig. 4l and m). We then constructed plasmids with KBS1 mutation and KBS2 deletion in the LGR5 promoter and found that neither knockdown nor overexpression of CBX8 affected the reporter gene activity (Fig. 4 l and m). These results suggest that in CC cells, CBX8 recruits KMT2b to KBS1 and KBS2 (also referred to as CBS2 and CBS4, respectively), promoting LGR5 transcription through H3K4me3.

RETRACTED

To identify the binding domain for CBX8 binding with KMT2b, we cloned five Flag-tagged CBX8 constructs (Fig. 4n) and transfected DLD-1 cells with the truncated plasmids. IP was performed on the cell extracts with anti-Flag antibodies. Flag-CB4 interacted with KMT2b in cancer cells (Fig. 4o), suggesting that the CBX8 domain between amino acids 214 and 300 is required for the interaction with KMT2b.

### Mettl3-induced m^6^A modification is involved in the upregulation of CBX8

The mechanism leading to aberrant expression of CBX8 is unknown. Previous studies have reported that m^6^A modification modulates all stages of the RNA life cycle and thereby regulates the expression and functions of RNAs [16, 17]. RMBase (http://rna.sysu.edu.cn/rmbase/index.php) prediction revealed that numerous m6A sites with very high confidence are distributed in CBX8 mRNA, so we elucidated whether upregulation of CBX8 is dependent on m^6^A modification. m^6^A RNA IP (RIP) combined with qRT-PCR revealed that m^6^A was significantly more enriched in DLD-1 and SW480 cells than in normal NCM460 cells (Fig. 5a). Given that Methyltransferase-like 3 (Mettl3) is the key m^6^A methyltransferase (“writer”) in mammalian cells, we evaluated Mettl3 expression and the correlation between Mettl3 and CBX8 expression in the TCGA database. Notably, Mettl3 was significantly upregulated in CC tissues, and Mettl3 expression was positively correlated with CBX8 expression (R = 0.53, Fig. 5b, c). Additionally, we silenced and upregulated Mettl3 with Mettl3 siRNAs and overexpression plasmids, respectively. Mettl3 depletion apparently reduced CBX8 mRNA and protein levels (Fig. 5d; Additional file 6: Figure S6A). In contrast, overexpression of Mettl3 increased mRNA and CBX8 protein levels (Fig. 5e; Additional file 6: Figure S6B). RIP assays also revealed that silencing Mettl3 reduced m6A modification of CBX8 mRNA in DLD-1 cells (Fig. 5f). Furthermore, we assessed the CBX8 mRNA stability in CC cells upon Mettl3 inhibition or overexpression. After treating cells with actinomycin D to block the de novo synthesis of RNA, the depletion of Mettl3 resulted in a decreased stability of CBX8 mRNA (Fig. 5g), whereas, overexpression of Mettl3 could increase the stability of CBX8 mRNA (Fig. 5g). Revealing that Mettl3, the m^6^A writer, specifically maintains the stability of CBX8 mRNA by promoting m^6^A modification in CC cells.

**Fig. 5:** Mettl3-induced m^6^A modification is involved in the upregulation of CBX8. **a,** RIP-qPCR showing the stronger enrichment of m^6^A in DLD-1 and SW480 cells than that in NCM460 cells. **b,** Mettl3 expression was assessed using data from the TCGA. **C,** CBX8 expression was positively correlated with Mettl3 expression in an analysis of TCGA data. **d-e,** Western blot of Mettl3 and CBX8 after Mettl3 inhibition or overexpression in DLD-1 cells. **f,** RIP-qPCR showing the enrichment of m^6^A in DLD-1 after Mettl3 depletion. **g,** The decay rate of CBX8 mRNA after treatment with 2.5 μM actinomycin D for indicated times, with Mettl3 knockdown or overexpression in DLD-1 cells. **h,** RIP-qPCR showing the enrichment of IGF2BP1 on CBX8 mRNA in DLD-1 and SW480 cells. **i,** Western blot of IGF2BP1 and CBX8 after IGF2BP1 inhibition in DLD-1 cells. **j,** The decay rate of CBX8 mRNA after treatment with 2.5 μM actinomycin D for indicated times, with IGF2BP1 knockdown in DLD-1 cells. **k,** RIP-qPCR showing the enrichment of IGF2BP1 on CBX8 mRNA in DLD-1 with Mettl3 knockdown. **l,** The schematic figure shows that mettl3 upregulates m^6^A level of CBX8 mRNA, IGF2BP1 binding to m^6^A sites to sustain the stability of CBX8 mRNA; CBX8 overexpression recruits KMT2b and Pol II to activate LGR5 by inducing H3K4me3, which regulates cancer stemness and chemosensitivity in CC. The relative enrichment in the RIP-qPCR assay was normalized by input. Data are shown as the mean ± SD of three replicates (*, *P* < 0.05; **, *P* < 0.01)

Then, we explored the mechanism involved in the Mettl3-induced stability of CBX8 in CC cells. Insulin-like growth factor 2 mRNA-binding protein 1 (IGF2BP1), a “reader” of m^6^A, plays a specific role in controlling the stability of m^6^A modified mRNA [18]. We predicted the potential readers of CBX8 m^6^A sites with RMBase and found that IGF2BP1 indeed has binding sites on CBX8 mRNA. A RIP assay confirmed the existence of a direct interaction between IGF2BP1 and CBX8 mRNA in CC cells (Fig. 5h). Silencing IGF2BP1 in DLD-1 cells significantly decreased CBX8 protein levels (Fig. 5i). After treating cells with actinomycin D, the median half-life of CBX8 mRNA was significantly reduced upon IGF2BP1 depletion (Fig. 5j). In addition, the interaction between IGF2BP1 and CBX8 mRNA was impaired after Mettl3 suppression (Fig. 5k). Taken together, our data suggest that IGF2BP1 binds to CBX6 mRNA to enhance its stability in an m^6^A-dependent manner. The schematic of Fig. 5l showed the mechanism of m^6^A-induced CBX8 regulating CC stemness.

RETRACTED

### Clinical relevance of the Mettl3/CBX8/LGR5 axis in CCs

Analyses of TCGA and GTEx data demonstrated that CC tissues had significantly higher levels of CBX8 expression than normal tissues (*P* < 0.01, Additional file 1: Figure S1A). This trend was further verified in randomly selected specimens by qRT-PCR and Western blotting (Fig. 6a-b). In addition, the IHC results confirmed that the high CBX8 expression was mainly located in cell nuclei in CC tissues (Fig. 6c). To further evaluate the relationship between CBX8 and chemosensitivity, we examined CBX8 expression in CC tissues and chemoresistant CC tissues via Western blotting. CBX8 expression was higher in chemoresistant CC tissues than in chemosensitive CC tissues (Fig. 6f). Then, we evaluated the potential correlation between CBX8 expression and patient outcome based on 283 cases with prognostic data from TCGA. Kaplan-Meier analysis revealed that higher expression of CBX8 was associated with lower disease-free survival rates (*P* = 0.048, Fig. 6d) but not with lower overall survival rates (*P* = 0.63, Fig. 6e).

**Fig. 6:** Clinical relevance of the Mettl3/CBX8/LGR5 axis in CC. **a,** The relative expression levels of CBX8 were assessed by qRT-PCR in 18 paired normal tissues and CC tissues. **b,** The protein expression of CBX8 was assessed by Western blotting in 6 paired normal tissues and CC tissues. **c,** The expression of CBX8 in normal tissues and CC tissues was assessed by IHC. **d,** The graph shows the results of Kaplan-Meier analysis of the disease-free survival (DFS) rate in CC patients in the TCGA database with high or low expression of CBX8. **e,** The graph shows the results of Kaplan-Meier analysis of the overall survival (OS) rate in CC patients with high or low expression of CBX8. **f,** The protein expression of CBX8 was assessed by Western blot in chemoresistant CC tissues (R1–6) and chemosensitive CC tissues (S1–6). **g,** Patients with chemoresistance had higher levels of CBX8, Mettl3, LGR5, CD133 and CD44 expression as assessed by IHC, while patients with chemosensitivity had relatively lower levels of CBX8, Mettl3, LGR5, CD133 and CD44 expression as assessed by IHC. **h,** The graph shows that CBX8 expression was positively correlated with LGR5, CD133, CD44 and EpCAM expression in an analysis of TCGA data. Data are shown as the mean ± SD of three replicates (*, *P* < 0.05; **, *P* < 0.01)

We further investigated the relationships among CBX8, Mettl3, LGR5 and stemness markers in patients with CC. As shown in Fig. 6g, patients with chemoresistance had higher levels of CBX8, Mettl3, LGR5, CD133 and CD44 expression than patients with chemosensitivity. In addition, dot plot analyses of TCGA datasets showed that the expression of CBX8 was positively correlated with the expression of Mettl3 (R = 0.53, *P* = 0.000), LGR5 (R = 0.34, P = 0.000), CD133 (R = 0.24, P = 0.000), CD44 (R = 0.34, P = 0.000) and EpCAM (R = 0.45, P = 0.000) in CC tissues (Fig. 6h, Fig. 5c).

RETRACTED

## Discussion

CSCs have intrinsic chemoresistant properties and can be selectively enriched during chemotherapy, ultimately resulting in chemotherapy failure and cancer recurrence [19]. The CBX protein family includes CBX2, CBX4, CBX6, CBX7 and CBX8, and CBX proteins have been reported to be associated with stemness properties and chemosensitivity. For instance, overexpression of CBX7 enhances self-renewal of hematopoietic stem cells (HSCs) and induces leukemia [20]. In addition, CBX7 is associated with tamoxifen sensitivity and chemosensitivity in breast tumors, whereas CBX2 has been found to be associated with chemoresistance [21]. The above findings suggest that CBX proteins may play vital roles in the regulation of stemness properties and chemosensitivity. Our study revealed that CBX8 was significantly overexpressed in chemoresistant CC tissues and positively correlated with the expression of stemness markers such as LGR5, CD133 and CD44 in CC tissues. Depletion of CBX8 suppressed spheroid formation ability and stemness marker expression and enhanced the sensitivity of CC cells to L-OHP and CPT-11, suggesting that CBX8 is an important regulator of stemness and a potentially good marker for predicting chemosensitivity in CC. We also examined the relationship between CBX8 expression and the prognosis of CC patients using data from the TCGA database. CBX8 expression negatively correlated with the RFS of CC patients. In addition, higher CBX8 expression tended to decrease OS, but this trend was not significant, perhaps due to the insufficient sample size in the TCGA database or the development of effective therapies for recurrent tumors in the last few years.

RETRACTED

CSC marker are essential for maintaining stemness properties, LGR5 belongs to the family of G protein-coupled receptors, was initially identified as a marker of intestinal stem cells [22]. Subsequent studies demonstrated LGR5+ stem cells were the origin of cancer in the intestine and LGR5 had been widely accepted as an ideal CSC marker of colorectal cancer [23–25]. According to the CSC concept, CSCs possess drug-resistant properties. LGR5 also conferred resistance to chemotherapeutic agents such as 5-Fu, oxaliplatin and irinotecan in CRC [10, 26, 27]. In our study, we isolated LGR5+ cells from CC cell line and confirmed that LGR5+ CC cells possessed stronger stemness properties and weaker sensitivity to chemotherapy. These results supported the notion that LGR5 was widely accepted CSC marker.

CBX8 has been reported to bind to H3K4me3 or H3K27me3 at the promoters of target genes to regulate transcription [5, 13]; H3K27me3, which is always bound by PRC1 complexes, marks transcriptional repression, while H3K4me3 marks transcriptional activation. Our data indicate that CBX8 loss decreases H3K4me3 at the promoter of LGR5 without changing H3K27me3, suggesting that CBX8 activates LGR5 through H3K4me3 modification in the promoter region. CBX8 is an essential component of the PRC1 complex, which comprises four subunits: a Ring E3 ubiquitin ligase subunit (RING1A/B), a Polyhomeotic subunit, a Posterior sex comb subunit, and a Polycomb subunit (CBX2, CBX4, CBX6, CBX7 or CBX8) [28]. The canonical function of CBX8 is believed to be essential for the recruitment of PRC1 to H3K27me3-modified genomic loci and subsequent repression of gene transcription [9]. For example, as a PRC1 component, CBX8 inhibits the expression of INK4a/ARF in fibroblasts to bypass cell senescence [29]. In our study, we discovered that CBX8 can sustain rather than suppress LGR5 expression by maintaining the transcription-activating histone modification H3K4me3. In addition, knockdown of Ring1b, an integral PRC1 component, failed to interfere with the expression of LGR5. These results suggest that CBX8 can activate LGR5 expression in a noncanonical PRC1-independent fashion. However, CBX8 cannot act independently; rather, it has been reported that CBX8 can associate with protein complexes to play noncanonical roles in transcriptional regulation. For instance, CBX8 recruits non-PRC1 complexes containing WDR5 to Notch network gene promoters to regulate Notch signaling, promoting breast tumorigenesis [5]. Therefore, we sought to identify any proteins involved in CBX8-mediated activation of LGR5 transcription, using an RNAi screening approach to identify potential H3K4 modifiers responsible for LGR5 regulation. Interestingly, we found that KMT2b physically regulates LGR5.

RETRACTED

KMT2b encodes a ubiquitously expressed lysine methyltransferase specifically responsible for the deposition of H3K4me3 at gene promoters [15, 30], which is required for embryonic stem cell development [15] and neuronal differentiation [31]. However, the role of KMT2b in cancers has rarely been documented. In our study, we discovered that CBX8 recruits KMT2b to the LGR5 promoter to maintain H3K4me3 modification status, implying that KMT2b potentially functions in tumorigenesis and tumor progression. Moreover, in stem cells, the classic function of KMT2b is to attach H3K4me3 to bivalent promoters with the aid of PRC1 component [15]; Interestingly, we found that the promoter of LGR5 which accumulated H3K4me3 and H3K27me3 was bivalent promoter. In addition, CBX8 is also a component of PRC1 complex. These results suggest that KMT2b exhibits classic functions in the bivalent promoter of LGR5. These results also imply that the PRC1-related bivalent mechanism of KMT2b exists not only in stem cells but also in solid tumors.

Aberrantly high expression of CBX8 has been identified in various tumors, but the underlying mechanism was unclear. m^6^A modification is an important epigenetic regulatory mechanism and is reported to influence alternative polyadenylation, pre-mRNA splicing, RNA stability and translation efficiency [32]. Mettl3 is a key member of the m^6^A methyltransferase complex and functions as the m^6^A “writers”. It is reported that Mettl3 sustained mRNA stabilization of SOX2 in m^6^A-dependent manner to persist stem-like phenotype and prevent radiation-induced cytotoxicity in glioma [33] and CRC [32]. We demonstrated that m^6^A modification induced by Mettl3 could sustain the stability of CBX8 mRNA, thus, promoting stemness and attenuating chemosensitivity. Our results provided complementary mechanism regarding mettl3-mediated stemness regulation. m^6^A modification exerts biological functions by binding to the m^6^A “reader”, including IGF2BP1 [34]. IGF2BP1 recognize the consensus GG(m^6^A) C sequence through the K homology domains, and enhance the stability and translation of their target mRNAs in an m^6^A-dependent manner [18]. Here, we also demonstrated that IGF2BP1 bind directly to CBX8 mRNA and promote CBX8 expression in an m^6^A-dependent manner, which was consistent with previous findings.

RETRACTED

In summary, we have demonstrated that CBX8 is a master regulator of cancer stemness and chemosensitivity in CC. More importantly, CBX8 can recruit KMT2b and Pol II to the LGR5 promoter to maintain H3K4me3 status and thus promote LGR5 expression. Furthermore, aberrantly overexpression of CBX8 was induced by Mettl3-mediated m^6^A modification. Our findings not only reveal the mechanism by which CBX8 regulates stemness but also provide potential new therapeutic targets to overcome the chemoresistance of CC.

## Conclusions

CBX8 can maintain the stemness and inhibit the chemosensitivity of CC in vivo and in vitro. Mechanistically, noncanonical CBX8 recruited KMT2b and Pol II to the LGR5 promoter to promote its expression by maintaining the histone H3K4me3 status. Aberrant overexpression of CBX8 was induced by Mettl3-mediated m^6^A modification. This study provides useful therapeutic targets for reversing stemness and enhancing chemosensitivity.

## Supplementary information

**Additional file 1: Figure S1.** CBX proteins expression are examined in public database or CC tissues. **A,** CBX proteins expression were assessed using data from the TCGA and GTEx databases. **B,** The expression of CBX2, CBX4 and CBX8 was assessed by IHC scores in 20 chemoresistant CC tissues and 20 chemosensitive CC tissues. Data are shown as the mean ± SD of three replicates (*, *P* < 0.05; **, *P* < 0.01).

**Additional file 2: Figure S2.** The effects of CBX8 on CC stemness. **A,** CBX8 mRNA expression in 8 different cell lines. **B**, The incidence of tumor formation was shown in the chart. **C,** DLD-1 cells with or without CBX8 depletion were injected into the subcutaneous tissues of nude mice at a density of 5 × 10^4^, 1 × 10^4^, 1 × 10^3^ or 1 × 10^2^ cells per mouse. 40 days later, the number of mice that had developed tumours was counted. The frequency of CSC cells was calculated using ELDA software. **D,** The expression of CBX8 and CSC markers was examined by qRT-PCR in sorted LGR5+ and LGR5- cells. **E,** number of sphere formation in sorted LGR5+ and LGR5- cells. **F-G,** The relative expression of CBX8 and LGR5 was detected by qRT-PCR in CC cells with CBX8 knockdown or overexpression. Data are shown as the mean ± SD of three replicates (*, *P* < 0.05; **, *P* < 0.01).

RETRACTED

**Additional file 3: Figure S3.** Determination of additive or synergistic effects on cell colony formation and apoptosis. **A.** Determination of additive or synergistic effects on cell colony formation. Additive effects on CC proliferation are indicated by the sum of the individual effects of CBX8 depletion or overexpression and of L-OHP or CPT-11. Synergistic effects are indicated by the combined effects of silencing or overexpressing CBX8 in cells treated with L-OHP or CPT-11. The colony formation rate of shCtrl or vec DLD-1 cells was set to 100%. **B.** The determination of additive or synergistic effects on cell apoptosis. Data are shown as the mean ± SD (* *P* < 0.05; ** *P* < 0.01).

**Additional file 4: Figure S4.** CBX8 promotes CC stemness and inhibits chemosensitivity through LGR5. **A,** CBX8 was preferentially distributed near the TSS of genes. **B,** GO analysis of CBX8-binding genes. **C,** Primary and secondary sphere formation were assessed in CBX8-depleted DLD-1 cells with or without LGR5 overexpression, and in CBX8-overexpressing SW480 cells with or without shCBX8 transfection. **D,** The expression of CSC markers was examined by qRT-PCR in CBX8-depleted DLD-1 cells with or without LGR5 overexpression, or in CBX8-overexpressing SW480 cells with or without shCBX8 transfection. **E,** The apoptotic rate of CBX8-depleted DLD-1 cells with or without LGR5 overexpression, or CBX8-overexpressing SW480 cells with or without shCBX8 transfection after treatment with L-OHP or CPT-11 at the concentrations of 10 μmol/L. Data are shown as the mean ± SD of three replicates (*, *P* < 0.05; **, *P* < 0.01).

**Additional file 5: Figure S5.** The enrichments of Pol II, H3K27me3 or H3K27Ac are detected in CC cells with CBX8 overexpression or knockdown. **A,** ChIP-qPCR analysis was used to assess the binding affinity of Pol II to the CBS1-CBS4 regions after CBX8 overexpression in DLD-1 cells. **B-C,** ChIP-qPCR analysis identified the enrichment of H3K27Ac and H3K27me3 in the CBS1-CBS4 regions after CBX8 knockdown in DLD-1 cells. Data are shown as the mean ± SD of three replicates (*, *P* < 0.05; **, *P* < 0.01).

**Additional file 6: Figure S6.** Mettl3 changes the mRNA expression of CBX8. **A-B,** the mRNA level of Mettl3 and CBX8 were examined after Mettl3 knocked down or overexpression. Data are shown as the mean ± SD of three replicates (*, *P* < 0.05; **, *P* < 0.01).

**Additional file 7.** Supplemental Methods

## Data Availability

The datasets used and/or analysed during the current study are available from the corresponding author on reasonable request.

## Abbreviations

ATCC: American Type Culture Collection
CC: Colon cancer
ChIP: Chromatin immunoprecipitation
CPT-11: Irinotecan
CRC: Colorectal cancer
CSC: Cancer stem cell
DEAB: Diethylaminobenzaldehyde
GO: Gene ontology
GSEA: Gene set enrichment analysis
GTEx: Genotype-tissue expression
HCC: Hepatocellular carcinoma
IHC: Immunohistochemistry
IP: Immunoprecipitation
L-OHP: Oxaliplatin
PRC1: Polycomb repressive complex 1
TCGA: The Cancer Genome Atlas
